# *FVC-NET*: An Automated Diagnosis of Pulmonary Fibrosis Progression Prediction Using Honeycombing and Deep Learning

This article has been retracted.

**DOI:** 10.1155/2022/2832400

**Published:** 2022-01-28

**Authors:** Anju Yadav, Rahul Saxena, Aayush Kumar, Tarandeep Singh Walia, Atef Zaguia, S. M. Mostafa Kamal

**Affiliations:** ^1^Manipal University Jaipur, Jaipur, India; ^2^School of Computer Application, Lovely Professional University, Phagwara, India; ^3^Department of Computer Science, College of Computers and Information Technology, Taif University, Taif 21944, Saudi Arabia; ^4^Department of Mathematics, Islamic University, Kushtia 7003, Bangladesh

## Abstract

Pulmonary fibrosis is a severe chronic lung disease that causes irreversible scarring in the tissues of the lungs, which results in the loss of lung capacity. The Forced Vital Capacity (*FVC*) of the patient is an interesting measure to investigate this disease to have the prognosis of the disease. This paper proposes a deep learning-based *FVC-Net* architecture to predict the progression of the disease from the patient's computed tomography (CT) scan and the patient's metadata. The input to the model combines the *image score* generated based on the degree of honeycombing for a patient identified based on segmented lung images and the metadata. This input is then fed to a 3-layer net to obtain the final output. The performance of the proposed *FVC-Net* model is compared with various contemporary state-of-the-art deep learning-based models, which are available on a cohort from the pulmonary fibrosis progression dataset. The model showcased significant improvement in the performance over other models for modified Laplace Log-Likelihood (−6.64). Finally, the paper concludes with some prospects to be explored in the proposed study.

## 1. Introduction

Interstitial lung disease (ILD) is a term for a cluster of conditions comprising Idiopathic Pulmonary Fibrosis (IPF) [1]. Fibrotic ILD such as IPF is exemplified by fibrotic destruction of the lung parenchyma concerning medical performance and prediction. IPF is an intensifying fibrotic lung disease linked with a desolate prognosis and an average survival of around three years [2]. However, in clinical practice, the path of the disease in specific patients may fluctuate significantly. Pulmonary fibrosis is a progressive disease that usually degrades over time. This degradation is known as the extent of fibrosis which is the scarring inside the lungs [2]. Patients with this disease experience the evolution of fibrosis at vastly different rates. Some patients develop the scarring slowly and bear with the disease for several years, whereas others deteriorate more quickly, leading to death [3]. When scarring occurs, the patient finds it difficult to breathe normally, which eventually leads to shortness of breath even when the person is not performing any strenuous exercise [4]. Patients with this disease display fibrotic sections, honeycombing, and wide-ranging patchy ground-glass areas with or without consolidations, depicting the presence of pleural fluid within the CT scans [5]. Hence, biomedical imageries are a massive source of knowledge beneficial to feed analytical tools within revealing pathologies [6]. But due to the extreme unpredictability of this disease, it becomes a challenging task even for qualified radiologists, further making it even harder for the doctors to determine the prognosis in patients with IPF.

The evolution of the disease in Idiopathic Pulmonary Fibrosis (IPF) is assessed by the decrease in Forced Vital Capacity (FVC) [7]. FVC is a measurement used to determine the lung function of the patients; it is measured by an instrument called a spirometer, which measures the amount of air inhaled and then exhaled [8]. Forced Vital Capacity (FVC) has been proved as the most efficient magnitude for years to evaluate and gather information about the functional status of patients with fibrotic lung diseases; a deterioration of FVC is considered as a sign of progression of the disease. Despite dependable tendencies of FVC deterioration in the pulmonary fibrosis patients, the trend of the progression in patients is not very predictable, and significant variability in FVC is detected over time [7].

Many machine learning and deep learning models have been developed to determine the possibility of IPF by using the CT images of lungs. This made the detection much easier for the doctors. Most of the methods proposed in the literature have considered a full set of CT images whereas we have used two random images of one patient to calculate the IPF. However, there are very few machine learning models to predict the progression of this disease precisely and accurately. In light of this statement, the *contribution of the paper can be written as follows:*

1. An efficient model is proposed for *computed tomography* images that can diagnose human lungs with Idiopathic Pulmonary Fibrosis and then integrate it with the patient's metadata which allows us to find the patient's decline in FVC in the forthcoming weeks
2. This model can be used to calculate the rate of FVC decline that can be correlated with the speed of survival of the patient
3. The proposed model results are compared with the current state-of-the-art methods over the same metrics

The remainder of the paper is organized as follows: Section 2 highlights state-of-the-art methods over the disease and the techniques utilized to measure the FVC decline.  Section 3 explains the proposed methodology and FVC-Net architecture in detail.  Section 4 presents the results using the proposed architecture. Further, a comparative analysis is shown with other methods and techniques over the problem.  Section 5 justifies the applicability and validity of the proposed FVC-Net model on a different scenario *(COVID-19 case study)*. Finally, Section 6 concludes the paper with future directions to the work.

## 2. Related Work

This section surveys the methods and techniques for identifying the disease based on the FVC decline. In the preliminary investigations, Kim DS et al. did research that evidenced that the deterioration in FVC over 6 to 12 months has been dependably connected with a declined survival rate. They also concluded that when the FVC drop is in the range of 5 to 10%, the predictive chances of mortality are high. King TE Jr et al. [3] verified that the baseline FVC is of uncertain predictive value. This claim was also supported by Jegal and others in their contribution [10].

Raghu et al. [11] characterized that IPF has an unpredictable deterioration in the patients' lung capacity, and it disturbs the aged crowd typically, mainly in the age group of 50 to 70 years. They also found that the median survival period was 3.8 years through the period 2001 to 2011. Raghu et al. did a study that demonstrates that smoking, environmental exposure, and microbial agents act as risk factors. They also studied the indications of this disease, primarily respiratory such as dry cough, fatigue, shortness of breath, reduced pulmonary function test results, and finally patterns of fibrosis in CT images of lungs [12].

Zappala et al. concluded that even more minor, i.e., 5–10%, and sustained changes in Forced Vital Capacity can represent disease progression [13]. Raghu et al. proposed that maximum patients with IPF demonstrate a steady deterioration of lung function over the years. A minority of patients remain stable or deteriorate rapidly [14].

Lynch et al. explained that the features of CT scan images, such as fibrosis (scarring) and honeycombing, are powerfully associated with FVC measurements [3]. Flaherty et al. demonstrated that the patient's degree of scarring and honeycombing on CT scans are an extrapolative measure of their survival in pulmonary fibrosis [15]. Arabi et al. have shown that the CT scans images contain a lot of information for detecting various lung diseases [16]. In literature, various lung diseases related to fibrosis are detected from the honeycomb structures formed in the lungs. James [17] described the degree of honeycombing. It represents a pattern existing in the lung's CT image, categorized by small cystic airspaces, ranging up to several centimeters at times. Zrimec and Wong [18] described the cystic airspaces of the honeycomb structures and showed that they have dense fibrous tissue with thickened walls. It is also seen in the lung images of patients with IPF and pneumonia.

Comelli et al. proposed a quick and accurate lung segmentation method using a dataset of patients with IPF. They investigated two models: U-Net and E-Net. They concluded that E-Net is a better choice among the two as it produced comparatively fast (20.32 s) and accurate (dice similarity coefficient = 95.90%) results, and therefore, these models can be used to segment the lungs of patients and help achieve user-independent results, without the assistance of radiologists [7].

Walsh et al. performed a case study on deep learning methods for classifying scarring in lungs using CT images. They deduced that this method is highly cost-effective with good accuracy of about 76·4%, almost equivalent to human accuracy [15]. Kido et al. used algorithms like fully convolutional network (FCN), Lung nodule, R-CNN, Residual U-Net, U-Net, and V-Net and deduced that using DL, computer-aided diagnosis, is going to be much easier and more accurate than even an experienced radiologist; not just IPF, various other lung abnormalities can be detected using DL [5].

From literature, it has been observed that % FVC decline predictions play a vital role in patients' early prognosis and survival. Only a few authors studied the forecast of FVC decline in pulmonary fibrosis patients [19, 20]. These authors also have worked on pulmonary fibrosis progression challenge Kaggle 2020. But both the authors have not considered honeycombing for their findings. Also, it is found that the existing models suffer from overfitting [24, 25], poor convergence speed [26, 27], data misbalancing [28, 29], poor visibility [30, 31], and multiple light sources [32], etc. kind of problems. Therefore, in this paper, FVC-Net is proposed to overcome these kinds of problems.

## 3. Proposed Methodology

This section discusses the proposed methodology chosen to construct a deep learning model to predict the trends in the *FVC* of the patients. This section concentrates on the discussion over the (i) *dataset description* and (ii) *proposed model for FVC-Net.*

### 3.1. Dataset Description

To train our model, a dataset from *Kaggle* [9] has been utilized. The dataset contains CSV metadata along with the CT scans for each patient. The metadata contains 1549 rows and seven columns with the fields *Patient's ID, Percent, Age, FVC, Sex, Weeks,* and *Smoking Status*. The CT scans for each patient were available to us in individual folders named according to the patient's ID. Each folder contained the CT scans of the patient. It is noted as week 0. Accordingly, their *FVC* measurement has been indicated in terms of week number for one to two years. We have been provided with early measurements of the *FVC* and the scans. The sample stack of CT scan images of a patient is shown in Figure 1.

### 3.2. Proposed Model FVC-Net

In this section, the proposed model is explained for the prediction of *FVC* over pulmonary fibrosis progression. The dataset contains two major parts. One is the patient's demographic data (*Patient*'*s ID, Percent, Age, FVC, Sex, Weeks,* and *Smoking Status*) and their CT images. We have analyzed that metadata also plays a vital role in the prediction of pulmonary fibrosis progression. The proposed model *FVC-Net* has three stages. *Stage 1* is image preprocessing, *Stage 2* is metadata formation, and *Stage 3* is to design the *FVC-Net* model. The proposed methodology is explained in Figure 2.

FVC of the patient can be predicted using the initial slope of FVC of that patient. First CT scans are preprocessed, *CT* ∈ *ct*_*i*_, *ct*_*i*+1_, *ct*_*i*+2_,…, *ct*_*n*_, where *n* represents the number of patients. Each CT scan contains multiple slices of lungs, i.e., *ct*_*i*_ ∈ {*S*_1_, *S*_2_, *S*_3_,…, *S*_*n*_}; we randomly selected two slices *S*_*k*1_ and *S*_*k*2_ from *ct*_*i*_ for the feature extraction, where *i* is the number of slices and *k*1 and *k*2 are an index of the slice selected. The selected slices *S*_*k*1_ and *S*_*k*2_ are taken as input for FVC-Net model for extraction of CT features. Finally, metadata is formed by concatenating demographic data of each patient and their degree of honeycombing (i.e., image score) as feature set *M* ∈ {*M*_1_, *M*_2_, *M*_3_,…, *M*_*n*_} where *n* is a number of patients. Finally, both the feature sets are used to predict the slope of FVC, *SL* ∈ {*sl*_*i*_, *sl*_*i*+1_, *sl*_*i*+2_,…, *sl*_*n*_}. Every patient has FVC values *sl*_*i*_ ∈ {*FVC*_*we*_1__, *FVC*_*we*_2__, *FVC*_*we*_3__,…, *FVC*_*we*_*n*__}, where e_n is number of *FVC* values and *w* is week number.

FVC can be written for *n*^th^ patient in the *l*^th ^ week as

(1) $$\begin{array}{c} FVC_{we_{l}}={\text{slope}}_{n}*we_{l}+FVC_{\text{base}}, \end{array}$$

where *FVC*_base_ is the *FVC* value given as base and *slope*_*n*_ is the slope of *n*^th^ patient.

#### 3.2.1. Image Preprocessing

In this, the first step would be to preprocess the given DICOM images and then segment just the lung portion from the entire scan to obtain helpful information. The three crucial steps of image preprocessing are windowing, sampling, and segmentation.

 
*Windowing*. Windowing or grey-level mapping is a technique through which the greyscale component of the CT image is manipulated using the HU numbers. Doing this affects the look of the scan and accentuates the required structure (see Figure 3).
 
*Resampling*. Resampling implies changing the scale of an image. This can be done by changing the picture's pixel dimensions. Voxel size resampling was investigated to minimize the variability in feature values due to differing voxel sizes (see Figure 4).
 
*Segmentation*. Segmentation is an essential part of dealing with medical images, as it is used to extract the region of interest. The following stages were involved in the process of image segmentation: images were first *normalized*. Then, lungs were separated from the entire scan using the clustering technique (*K-Means).* Further, *thresholding* of the images was done to create a binary image. This separates the lung structure from background pixels to support the image processing (see Figure 5). In continuation to that, *morphology* was the following technique employed where the images were morphed using erosion and dilation, which are contraction and expansion, respectively. This was used to remove the undesired border areas and label different scan regions differently (see Figure 5) [5]. If the scan is denoted as a function of *x*, and the structuring function as another function, the grayscale *dilation* is shown as

(2) $$\begin{array}{c} \left(f\;⊕\;b\right)\left(x\right)=\sup_{y\in E}\left[f\left(y\right)+b\left(x-y\right)\right]. \end{array}$$

And the grayscale *erosion* is shown as

(3) $$\begin{array}{c} \left(f\;⊖\;b\right)\left(x\right)=\inf_{y\in B}\left[f\left(x+y\right)-b\left(y\right)\right]. \end{array}$$

Different regions of the CT scan are labeled differently with different colors. Finally, a *lung mask* is created using the steps mentioned above. This mask is then applied to the original image to obtain the final output, which is the segmented lung structure (see Figure 5).

#### 3.2.2. Finding the Degree of Honeycombing

After segmentation, the segmented images of the lungs are obtained for each patient. To calculate the degree of honeycombing, Sobel's edge detection is applied to the segmented lungs to find the edges of the images (white regions in the lungs). Further, the density of edges in the image is calculated, which gives us the degree of honeycombing. This process is repeated for every CT scan of a patient. And then, a mean score is calculated (degree of honeycombing) for that patient. This process is then repeated for each patient in the metadata. The Sobel's operator used for edge detection and D_E_, degree of honeycombing, is discussed in detail (see Figure 6).

The Sobel's operator uses two 3 × 3 kernels which are convoluted with the *S*_*k*1_ and *S*_*k*2_ to evaluate estimates of the derivatives for horizontal changes and also for the vertical changes. If *S*_*k*1_ and *S*_*k*2_ are considered as a source image, and *G*_*x*_ and *G*_*y*_ are images that contain the horizontal and the vertical derivate at each point, the computations are done as follows:

(4) $$\begin{array}{c} G_{x}=\left[\begin{array}{ccc} +1 & 0 & -1\\ +2 & 0 & -2\\ +1 & 0 & -1 \end{array}\right]*A,\\ G_{y}=\left[\begin{array}{ccc} +1 & +2 & +1\\ 0 & 0 & 0\\ -1 & -2 & -1 \end{array}\right]*A. \end{array}$$

*∗*symbolizes the 2D signal processing convolution operation.

The degree of honeycombing is the number of edge pixels in the segmented lung scan after the edge detection step [16]. It is calculated as follows:

(5) $$\begin{array}{c} D_{E}=\frac{1}{N}\sum_{x}\sum_{y}E_{v}\left(x,y\right), \end{array}$$

where *E*_*v*_(*x*, *y*) is the extent of vertical edges at some spot (*x*, *y*) and *N* is the amount of non-zero vertical edge pixels in that specific spot.

#### 3.2.3. Metadata Preparation

The Kaggle dataset in consideration has metadata of the patients along with their CT scans of the lungs. There are 1549 rows and 7 columns. The information regarding each patient is as follows: *Patient, Weeks, FVC*, *Percent, Age*, *Sex,* and *Smoking Status.* The metadata is preprocessed for FVC-Net model; the following changes were made (see Table 1).

The “Sex” and “Smoking Status” columns have been changed into numerical values. Patient records having little or no data about them (kept patients with at least 3 readings of their FVC) have been dropped. The demographic data were first normalized using the formula $z^{\prime }=\left(\left(\;z\;-\;\bar{z}\right)/\sigma \right)$, where *z* is the numeric feature in dataset, $\;\bar{z}$ is the arithmetic mean, and *σ* is the standard deviation.

After calculating the degree of honeycombing, image scores are added to the metadata. Table 1 showcases the final patient data after combining the image score.

#### 3.2.4. FVC-Net Model Architecture

The architecture of the proposed model *FVC-Net* is shown in Figure 7. The CT scan images of the patient to be provided as input sizes are resized to 512-by-512-by-1 before feeding it into the model. The input to the model undergoes Conv. (convolution), BN (batch normalization), and ReLU (rectified linear unit) twice, followed by averagePooling2D to obtain a concatenated single branch of size 256-by-256-by-64. Similarly, this branch undergoes Conv., BN, and ReLU multiple times to reach a size of 64-by-64-by-128, after which GlobalAveragePooling2D is done to decrease the size to 128. A new third branch is used to input the patient's metadata. Both these branches are concatenated. The final two layers are dense and dropout layers with a persistent decline in depth. The total number of parameters is 1,809,653, in which 1,808,629 are trainable parameters and 1,024 are nontrainable parameters. The optimizer chosen is “Adaptive Moment Estimation” (Adam) to modify the attributes of the neural network like the learning rate or the weights to minimize the losses.

Let *S*_*k*1_ and *S*_*k*2_ be input slices of *ct*_*i*_ of patients such that *S*_*k*1_ and *S*_*k*2_ ∈ *R*^*p*×*q*×1^  (*p*, *q* are spatial dimension) for the given input *ct*_*i*_ images. *S*_*k*1_ and *S*_*k*2_ are used by the CNN to calculate the feature vector from the last layer *F*_fvc-net_∈*R*^*p*^1^×*q*^1^×1^. *F*_fvc-net_ is the final feature extracted from *S*_*k*1_ and *S*_*k*2_ CT images. *F*_*dh*_ will be the set of normalized features from demographics and the degree of honeycombing. Finally, *F*_fvc-net_ and *F*_*dh*_ are passed to a fully connected layer for calculation of slope (*slope*_*n*_) of FVC which is used to predict the decline. The FVC is computed as

(6) $$\begin{array}{c} FVC_{we_{l}}=slope_{n}*we_{l}+FVC_{\text{base}}, \end{array}$$

where the baseline *FVC* is represented by *FVC*_*base*_ and *l* as the index of the week.

## 4. Result Analysis

In this section, the prediction of lung decline progression in chest CT images due to pulmonary fibrosis has been evaluated by *FVC-Net*. Its result is compared with various standard models. To show the adequate performance of the model, the following evaluations are conducted.

First, the evaluation metric for training loss and validation loss performance is calculated for the proposed model, i.e., *FVC-Net*.

Secondly, predicted FVC decline by *FVC-Net* is compared with the EfficientNets (EN), EfficientNets with Quantile Regression (EQR), logistic regression (*LR*), and random forest (*RF*). Further, the %*FVC* decline comparison is graphically represented for *FVC-Net* and other standard models. Finally, the *FVC-Net* model performance is also compared with models proposed in the literature.

### 4.1. Quantitative Analysis of *FVC-Net*

The evaluation measures mean squared error (*MSE*), mean absolute percentage error (*MAPE*), and mean absolute error (*MAE*) are used to assess the performance (training loss and validation loss) of the proposed model (*FVC-Net*).

*MSE:* MSE is one of the most used metrics that compute squared difference between the forecasted value and the actual value, divided by the number of values (see equation (7)). Therefore, it is the average of squared errors and [33] it may be used as a good measure for the goodness of fit. It is given by the following formula:
  (7) $$\begin{array}{c} MSE=\frac{1}{N}\sum_{i=1}^{N}{\left(y_{i}-{\hat{y}}_{i}\right)}^{2}. \end{array}$$
*MAPE*: it is another popular metric for estimating the performance of the forecasted results (see equation (8)) [20]. It is given by the following formula:
  (8) $$\begin{array}{c} MAPE=\frac{1}{n}\sum_{t=1}^{n}\left|\frac{A_{t}-F_{t}}{A_{t}}\right|. \end{array}$$
Here, *A*_*t*_ refers to the actual value, whereas *F*_*t*_ is the value forecasted. “*t*” refers to the observation we are doing.
*MAE*: it is used to calculate closeness between the forecasts and actual results. MSE assigns more significant penalization to significant prediction errors, whereas MAE considers all errors as equivalent. Instead of calculating the sum of the square of errors, MAE uses the sum of the absolute value of error (see equation (9)) [21]. It is given by the following formula:
  (9) $$\begin{array}{c} MAE=\frac{1}{N}\sum_{i=1}^{N}\left|y_{i}-{\hat{y}}_{i}\right|. \end{array}$$

To assess the model performance, the training and validation loss *MSE*, *MAE*, and *MAPE* are considered. The optimum values are attained based on the hyper parameter settings*:* (i) *dropout* *=* *0.75* and (ii) *learning rate* *=* *0.003.* After rigorous hypertuning of parameters for training loss, *MSE, MAE,* and *MAPE* are 35.020, 4.2867, and 262.8361, respectively. And for validation loss, outstanding values for *MSE, MAE,* and *MAPE* are 43.0999, 5.1461, and 122.87, respectively (see Table 2). Further, to visualize the performance of the parameters *MSE, MAE,* and *MAPE,* plots are drawn for 100 epochs, dropout = 0.75 and learning rate = 0.0003 (see Figures 8–10). From Table 2, it is clearly seen that the proposed model performance is giving the best result for these hypertuned parameters.

### 4.2. *FVC-Net* Comparison with *EN*, *EQR*, *LR*, and *RF* for Predicted FVC

To measure the performance of the proposed model *FVC-Net*, a comparative analysis is done using the modified Laplace Log-likelihood score (MLL). Standard methods available in machine learning are considered for comparison, i.e., *EN*, *EQR*, *LR*, and *RF*. MLL score is always negative in value, and the higher score implies the better performance of the model for predicting pulmonary fibrosis progression.

All the models are evalu1ated based on an MLL as a metric with the same environmental setup. It is a helpful metric to consider when working with models predicting medical applications as it evaluates the models' confidence in their decisions. It reflects both the certainty of the prediction and the accuracy obtained. For each true *FVC* measurement, a confidence measure is also calculated, which is nothing but the standard deviation *σ* [20]. The metric is computed as follows:

(10) $$\begin{array}{c} \sigma_{clippe\;d}=\max\left(\sigma ,70\right),\\ △=min\left(\left|FVC_{true}-FVC_{predicted}\right|,1000\right),\\ metric=-\frac{\sqrt{2\;}△}{\sigma_{clipped}}-\ln\sqrt{2\;}\sigma_{clipped}\;\left(10\right) \end{array}$$

The error (Δ) is given a ceiling value of 1000 ml to prevent huge errors, negatively penalizing the results. In contrast, the confidence values (*σ*) are capped at 70 ml to signify the approximate measurement uncertainty in *FVC*. The MLL score is calculated for *FVC-Net, EN*, *EQR*, *LR*, and *RF* (see Table 3).

From Table 3, it is observed that the MLL score of *FVC-Net* surpasses *EN*, *EQR*, *LR*, and *RF*. Hence*, FVC-Net* proved to be the most optimal compared to the other two (see Table 3).

### 4.3. Percentage of FVC Decline Comparison Graphically between *FVC-Net*, *LR*, and *RF*

Pulmonary fibrosis affects everyone at different rates. Predicting the progression of the disease just by looking at the CT scans is a difficult task and makes the prognosis complicated. Using *FVC-Net*, we can expect the deterioration in *FVC* over any period. This is going to help the doctors significantly in determining the course of treatment. To analyze the performance of the model, two patients, *P1* and *P2*, are considered. To compare, those patients' data are taken whose *FVC* decline is given for some week.

And further, % *FVC* decline is calculated for the proposed model, i.e., *FVC-Net*, *LR*, and *RF*. To visualize the performance of the models, a graph is drawn for Patient *P1* with ID *ID00419637202311204720264, age* *=* *73, male, Ex-Smoker*, and *P2* with ID *ID00426637202313170790466, age* *=* *73, Male, Never Smoked*. From Figure 11, it is seen that the % *FVC* decline of *FVC-Net* (orange line) is very close to the original *FVC* (blue line) value at a particular week in comparison to LR (red line) and RF (green line) (see Figure 11).

In Figure 11, the *FVC-Net* predictions are very close to the original value for all the duration considered for evaluation. It shows that our models' performance surpasses all the other models' results and can predict the decline more accurately.

For better visualization, Table 4 is drawn. In Table 4, the predicted *FVC* value is computed from the initial *FVC* at week 50 for *FVC-Net*, and further, its comparison is shown with original, *LR*, and *RF*. From Table 4, it is observed that, for 50 weeks, for Patient *P1* original predicted *FVC* is 2756.4, and from *FVC-Net* *=* 2803, *LR* *=* 2650, and *RF* = 2855. Similarly, for Patient *P2*, the original predicted *FVC* is 2816.67, and from *FVC-Net* *=* 2884.29, *LR* = 2523.33, and *RF* = 2667. It can be clearly seen that the predictive *FVC* value of the proposed model *FVC-Net* is closer to the original predicted *FVC* value (see Table 4), which proves the performance of the model is better than others for clinical decisions.

### 4.4. Comparison of *FVC-Net* with the State-of-the-Art Models

The MLL score is used to find the pulmonary fibrosis progression for the proposed model, i.e., *FVC-Net*. Further, it is compared with methods proposed in the literature (see Table 5). It is observed that *FVC-Net* has the highest MLL score in comparison with other methods. *FVC-Net* achieved an MLL score of −6.6414, which is significantly higher than other available methods. MLL score value with Elastic Net Regression is −6.73, Ridge Regression −6.81, and Fibrosis Net −6.8188, which is most elevated than three winning solutions and Multiple Quantile Regression. From these results, it can be clearly seen that *FVC-Net*'s performance is better than other models. Evaluating pulmonary fibrosis progression through *FVC-Net* achieved a significantly good score and demonstrated the efficacy in constructing the deep neural network to support clinical decisions.

## 5. *FVC-Net* for Post-*COVID-19* Pulmonary Fibrosis Progression

IPF is a rare disease, but looking at the current pandemic situation due to the SARS-CoV-2, it has proven fatal. It can even lead to acute respiratory distress syndrome *(ARDS)* and pneumonia, which requires hospitalization [33, 34]. Studies have shown that lungs start developing fibrosis after four or more months of being hospitalized, especially when the patient is under a mechanical ventilator (more than 72%). Various mechanisms of respiratory injuries in *COVID-19* have been discovered, with both viral and immune-mediated mechanisms implicated [23]. Another follow-up study consisting of 24 patients started noticing features of pulmonary fibrosis after five weeks of discharge (in 62% of the cases). The persistent respiratory complications that arise from the *COVID-19* start causing significant long-term disability and even death due to the lung fibrosis progression. If these probable cases of pulmonary fibrosis after COVID-19 are detected in the earlier stages, it will make the prognosis much easier and may decrease the decline of lung function [21]. It was also found that there were significant differences in the degree or the intensity of pulmonary inflammation among patients with mild, moderate, and severe pulmonary fibrosis [22]. *FVC-Net* can be used to evaluate the patient's *CT* scan and the patient's metadata to predict the rate of *FVC* decline in the case of *COVID-19.*

## 6. Conclusions and Future Work

The proposed *FVC-Net* model used metadata and CT scan images to predict *FVC* and measured its performance through the modified Laplace Log-Likelihood score (−6.641). *FVC-Net* achieved a significant improvement compared to *EN*, *EQR*, *LR*, *RF,* and other models reported in the literature. The proposed method further states that high-resolution CT, evaluated by the proposed deep learning algorithm, provides a low-cost, fast, and accurate way to find the decline in the lung function of a patient suffering from pulmonary fibrosis. This method could be of great advantage to facilities where thoracic imaging expertise is inadequate to make prognosis for doctors easier. As future work, the model's performance can be assessed in the precise determination of the decline rate in FVC for COVID-19 affected patients. Further, a user interface can be created where the medical staff can upload the patient's FVC values, and the CT scans to study the trends in their FVC. This will make the prognosis less complex, and the doctors can find the most optimal way to treat the patients suffering from IPF.

## Figures and Tables

**Figure 1:** Stack of CT scan.

**Figure 2:** Proposed methodology of *FVC-Net* model for prediction of *FVC* in pulmonary fibrosis dataset.

**Figure 3:** Windowing (ID00264637202270643353440).

**Figure 4:** Resampling (ID00007637202177411956430) from 512 ∗ 512 to 334 ∗ 334.

**Figure 5:** Lung segmentation.

**Figure 6:** Edge detection. Patient ID ID00426637202313170790466 and its degree of honeycombing is 0.033362067.

**Figure 7:** Proposed model: FVC-Net architecture.

**Figure 8:** MSE-loss-100 epochs-D = 0.75.

**Figure 9:** MAE-loss-100 epochs-D = 0.75.

**Figure 10:** MAPE-loss-100 epochs-D = 0.75.

**Figure 11:** Comparison of the predictions from *FVC-Net* and LR and RF.

**Table 1:** Final metadata after adding degree of honeycombing.

Patients	Initial FVC	Age	Sex	Smoking status	Image score
ID00419637202311204720264	2920.15	73	Male	Ex-smoker	0.0024935
ID00422637202311677017371	1939.37	73	Male	Ex-smoker	0.015953544
ID00423637202312137826377	2771.34	72	Male	Ex-smoker	0.120674989
ID00426637202313170790466	3030.47	73	Male	Never smoked	0.033362067

**Table 2:** Training and validation loss

		Training			Validation		
Dropout	Learning rate	MSE	MAE	MAPE	MSE	MAE	MAPE
0.7	0.01	151.127	7.4348	597.8169	58.9223	5.5655	369.3281
0.7	0.001	49.6714	5.0131	393.4241	48.0598	5.2879	146.3218
0.7	0.003	40.8036	4.6676	347.9123	45.57	5.1772	187.84
0.7	0.0005	55.1239	5.258	282.2506	42.2396	4.7951	244.6641
0.75	0.01	247.2195	9.4761	972.0759	43.9481	4.3682	198.3117
0.75	0.001	53.3548	5.0557	316.7048	56.1926	5.9527	212.3215
***0.75 ***	***0.003***	***35.02***	***4.2867***	***262.8361***	***43.0999***	***5.1461***	***122.87***
0.75	0.0005	35.1473	4.294	406.3161	51.8677	5.4012	126.1631

**Table 3:** Results from different algorithms.

Algorithm	Score
FVC-Net	−6.641
EfficientNets with Quantile Regression	−6.8424
EfficientNets	−6.8855
Random forest	−7.3348
Logistic regression	−13.0544

**Table 4:** Comparison of the predictions from FVC-Net, LR, and RF

	Patient ID: ID00419637202311204720264				Patient ID: ID00426637202313170790466			
Model	Initial (FVC)	Time (weeks)	Predicted (FVC)	Slope	Initial FVC	Time (weeks)	Predicted (FVC)	Slope
*Original*	2920	50	2756.4	-3.271	3030	50	2816.67	−4.267
***FVC-Net***	**2920**	**50**	**2803**	−**2.34**	**3030**	**50**	**2884.29**	−**2.914**
*LR*	2920	50	2650	−5.4	3030	50	2523.33	−10.133
*RF*	2920	50	2855	−1.3	3030	50	2667	−7.26

**Table 5:** Comparison of Laplace Log-Likelihood scores for the proposed FVC-Net and other models in literature.

Comparison with different methods	Laplace Log-Likelihood
FVC-Net (proposed model)	−6.641
Elastic Net Regression [19]	−6.73
Ridge Regression [19]	−6.81
Fibrosis Net [20]	−6.8188
Kaggle 1st place [cf. 20]	−6.8305
Kaggle 2nd place [cf. 20]	−6.8311
Kaggle 3rd Place [cf. 20]	−6.8336
Multiple Quantile Regression [19]	−6.92

## Data Availability

The data used to support the findings of this study are available from the corresponding author upon request.
